The article "Assessing the Prognostic Performance of the Child-Pugh, Model for End-Stage Liver Disease, and Albumin-Bilirubin Scores in Patients with Decompensated Cirrhosis: A Large Asian Cohort from Gastroenterology Department" was retracted in 2023. Reasons: suspected computer-generated content; unreliable results or conclusions; concerns about the data; concerns about the results or conclusions.

# Assessing the Prognostic Performance of the Child-Pugh, Model for End-Stage Liver Disease, and Albumin-Bilirubin Scores in Patients with Decompensated Cirrhosis: A Large Asian Cohort from Gastroenterology Department

**DOI:** 10.1155/2020/5193028

**Published:** 2020-02-15

**Authors:** Si-Zhe Wan, Yuan Nie, Yue Zhang, Cong Liu, Xuan Zhu

**Affiliations:** Department of Gastroenterology, The First Affiliated Hospital of Nanchang University, Nanchang, Jiangxi, China

## Abstract

*Background and Aim*. Various methods, including the Child-Pugh score, the model for end-stage liver disease (MELD) score, the MELD combined with serum sodium concentration (MELD-Na) score, the integrated MELD (iMELD) score, and the albumin-bilirubin (ALBI) score, have been widely used for predicting the survival of decompensated cirrhosis (DeCi) patients. In this study, we defined and compared the prognostic value of these scores to predict mortality in DeCi patients.

**Methods:**

We performed a single-center, observational retrospective study and analyzed 456 DeCi patients who were hospitalized in the gastroenterology department. The biochemical examination results and demographic characteristics of the patients were obtained, and five scores were calculated upon admission after 24 hours. All patients were observed until death, loss to follow-up, or specific follow-up times (28 days, 90 days, and 6 months). A receiver operating characteristic (ROC) curve was used to evaluate the ability of these methods to predict mortality in DeCi patients.

**Results:**

At 28 days, 90 days, and 6 months, the cumulative number of deaths was 50 (11.0%), 76 (16.6%), and 91 (19.9%), respectively. The scores were significantly higher in nonsurviving patients than in surviving patients. All scores yielded viable values in predicting 28-day, 90-day, and 6-month prognoses for DeCi patients. The areas under the ROC curve (AUROCs) of the ALBI score were higher than those of the other scores, which were only over 0.700 at 28 days. The AUROC of the MELD score was higher than that of the other scores, including the MELD-Na and iMELD scores, at 90 days and 6 months.

**Conclusion:**

All five methods (Child-Pugh score, MELD score, MELD-Na score, iMELD score, and ALBI score) provided a reliable prediction of mortality for both the short-term and long-term prognosis of patients with DeCi. The ALBI score may be particularly useful for assessing short-term outcomes, whereas the MELD score may be particularly useful for assessing long-term outcomes.

## 1. Introduction

Liver cirrhosis has high morbidity and mortality and leads to a million deaths per year worldwide [1]. In Asia, hepatitis B virus (HBV) is the main cause of liver cirrhosis. Decompensated cirrhosis (DeCi) is one of the terminal liver diseases, which is often accompanied by different complications, including gastrointestinal variceal bleeding, infection, ascites, and hepatic encephalopathy (HE), among others [2–4]. Liver transplantation markedly improves survival in patients but is not widely available because of limited liver resources, high costs, and immunological transplantation [5]. Hepatic function is severely affected by patients' ability to work and quality of life. Economic burden caused by DeCi is still heavy. Patients with DeCi show significant differences in terms of survival and morbidity. Therefore, it is necessary to develop a simple and reliable prognostic method for determining the mortality risk in DeCi patients and help guide clinicians in therapeutic decision-making on the basis of the predictive outcomes.

Previous studies have shown the effectiveness of the Child-Pugh (CTP) score, the model for end-stage liver disease (MELD) score, and some modified MELD scoring systems [6–10]. The Child-Pugh score is determined by calculating serum bilirubin, albumin, prothrombin time, hepatic encephalopathy, and ascites [8]. It has been widely used in the clinic because of its simplicity since approximately 50 years ago. The MELD score is determined by three routine laboratory test results: bilirubin, creatinine, and international normalized ratio (INR), and it is by far the most commonly used method worldwide in the evaluation of patients for transplantation. However, in clinical practice, the MELD score does not include some important indicators that can reflect the prognosis of patients with DeCi, such as severe hyponatremia, age, and ascites. The adjusted MELD scores, including the MELD-Na score and the integrated MELD (iMELD) score, which include serum sodium and age, can evaluate the prognosis of patients with DeCi [11, 12]. Recently, a new, simple, and objective score—the albumin-bilirubin (ALBI) score—was used to assess liver function in DeCi patients, which is only calculated using albumin and bilirubin levels [13]. ALBI has proven to be an independent predictor of survival in patients with DeCi [14]. However, the study populations have been dominated by Caucasians in Europe and the United States, with mostly alcoholic liver cirrhosis. Nevertheless, all five methods (Child-Pugh score, MELD score, MELD-Na score, iMELD score, and ALBI score) are being used to a certain extent clinically. More studies are needed to define the prognosis predictions of the existing scores and find the most reliable method to predict prognosis in patients with DeCi, which is mainly caused by hepatitis B. To date, there are no data on the comparison of all five approaches in evaluating and predicting prognosis for DeCi patients. The aim of this study was to compare the short-term and long-term predictive significance and capacity of the Child-Pugh score, the MELD score, the MELD-Na score, the iMELD score, and the ALBI score for DeCi patients in China to guide clinical practice.

## 2. Patients and Methods

### 2.1. Study Design

This study was a retrospective long-term cohort study of patients admitted to a single center from January 2013 to December 2017. The study protocol was approved by the Institutional Ethics Committee of the First Affiliated Hospital of Nanchang University. Informed written consent was obtained from all the study participants.

### 2.2. Patients

All adult patients were admitted to the ward for decompensated cirrhosis. This cohort included all patients who were admitted for decompensated cirrhosis. Exclusion criteria included refusal to sign, pregnant women, cardiovascular disease, hematologic disorders, uremia, previous liver transplantation, and HIV infection. Survival was evaluated at 28 days, 90 days, and 6 months by direct phone calls and/or an assessment of medical records. All patients were treated following accepted recommendations and guidelines after admission to the hospital and were followed up until death or 6 months [15–17].

### 2.3. Definitions

Patients with DeCi were defined by clinical, biochemical, and radiological parameters, endoscopic results, the presence of ascites, hepatic encephalopathy (HE), and/or signs of portal hypertension, ultrasonography, and even histology [18]. The diagnosis of hepatorenal syndrome (HRS) and ascites is based on criteria proposed by the International Ascites Club and American Association for the Study of Liver Diseases (AASLD). Hepatic encephalopathy (HE) and acute-on-chronic liver failure were diagnosed according to West-Haven criteria, a well-established criterion defined by the Chronic Liver Failure (CLIF) Consortium [19, 20]. The Child-Pugh score was calculated according to TBIL, albumin, INR, ascites status, and degree of HE [8]. The MELD score was calculated according to the original formula: 3.8 × loge (bilirubin (mg/dl)) + 11.2 × loge (INR) + 9.6 × loge (creatinine (mg/dl)) + 6.4 × (etiology : 0 if cholestatic or alcoholic, 1 otherwise). The MELD-Na score was calculated by using MELD + 1.59 × (135 − Na (mmol/l)) [21]. The iMELD score was calculated by using MELD + 0.3 × age (years) − 0.7 × Na (mmol/l) + 10 [12]. The ALBI score was calculated by using 0.66 × log_10_(bilirubin (*μ*mol/l)) − 0.085 × (albumin (g/l)) [22].

### 2.4. Study Protocol

DeCi patients were included in the study at admission. During hospitalization, relevant demographics, medical history, clinical characteristics, presence of other comorbidities, etiology of cirrhosis, types of decompensation and number of complications, and blood test parameters at admission (such as routine blood tests, liver function test, and renal function test) were collected. The patients were followed up for 6 months to obtain survival information. Patients with incomplete follow-up at 28 days, 90 days, and 6 months were not included in the final analysis of the corresponding time. Considering the impact on the conclusion caused by patients with incomplete data, we compared the basic information and treatment differences between those who were lost to follow-up and the overall patient. Fortunately, no significant statistical differences were found. The information and treatment of patients who were lost to follow-up are shown in Supplementary [Supplementary-material supplementary-material-1].

### 2.5. Statistical Analysis

Statistical analyses were performed using SPSS software version 16.0 (SPSS Inc., Chicago, IL), and receiver operating characteristic (ROC) analysis was performed by using MedCalc statistical software version 15.2.1 (MedCalc, Ostend, Belgium). Continuous variables are described as the median (interquartile range (IQR)). Categorical variables are described as frequency (percentage (%)). Continuous variables were compared using the Mann-Whitney *U* test, and categorical variables were compared using the Chi-squared test or Fisher's exact test. The diagnostic accuracy of the prognosis score was tested by the receiver operating characteristic (ROC) curve, and the areas under the ROC curve (AUROCs) were compared using the DeLong test. Sensitivity and specificity were determined using the cut-off point with the highest Youden index (sensitivity + specificity − 1). All statistical tests were two-sided, and *P* < 0.05 was considered statistically significant.

## 3. Results

### 3.1. Sample Description

We studied a total of 456 patients with DeCi admitted to the hospital between January 2013 and December 2017. The median age (interquartile range) of the 456 patients was 53.5 (46-63.75) years (maximum 86 years and minimum 25 years). The majority of the patients were male (302/456, 74.6%). The demographic and biochemical characteristics of the study population are outlined in Table 1. The etiology of liver cirrhosis was hepatitis virus in 60.5% of patients (276/456), followed by alcoholic (15.8%, 72/456), cryptogenic cirrhosis (9.4%, 43/456), combined alcoholic with hepatitis virus (8.1%, 37/456), and other (6.1%, 28/456). The cause of decompensation events responsible for hospitalization was ascites (0.7%, 3/456), gastrointestinal hemorrhage (89.2%, 407/456), hepatic encephalopathy (4.8%, 22/456), and infection (5.3%, 24/456). The average length of hospital stay was 11 [9–13] days. A total of 64 (14.0%) patients received treatment in the intensive care unit (ICU), and 392 (86.0%) patients received treatment in the general ward. Twenty (4.4%) patients had renal failure, 56 (12.3%) patients had hepatocellular carcinoma, and 436 (95.5%) patients had acute decompensation. A total of 50 (11.0%), 76 (16.6%), and 91 (19.9%) patients died or accepted liver transplantation within 28 days, 90 days, and 6 months, respectively. The causes of death at 6 months were as follows: 15 (16.5%) patients had respiratory failure, 44 (48.4%) patients had hemorrhagic shock, 10 (11.0%) patients had hepatic encephalopathy, 5 (5.5%) patients had infectious shock, 5 (5.5%) patients had hepatorenal syndrome, 4 (4.4%) patients had liver failure, and 8 (8.8%) patients had an uncertain cause of death. The causes of death are summarized at 28 days, 90 days, and 6 months in Supplementary [Supplementary-material supplementary-material-1].

### 3.2. Comparison between the Survival Group and the Nonsurvival Group

The clinical laboratory characteristics and prognostic scores of the patients are listed in Table 2. DeCi patients were divided into nonsurviving and surviving groups according to their 28-day, 90-day, and 6-month outcomes. The AST, alkaline phosphatase (ALP), bilirubin, creatinine, gamma-glutamyl transpeptidase (GGT), INR, PTA, WBC, Child-Pugh score, MELD score, MELD-Na score, and iMELD score of the nonsurviving group were all significantly higher than those of the surviving group during any phase of the follow-up (*P* < 0.05), whereas the albumin of the nonsurviving group was significantly lower than that of the surviving group (*P* < 0.05). The ALT of the nonsurviving group was significantly higher than that of the surviving group at 6 months (*P* < 0.05), whereas the difference was not significant at 28 days or 90 days (*P* > 0.05). No significant differences in platelet or serum Na were observed at any follow-up time (*P* > 0.05).

### 3.3. Predictive Significance and Capacity of the Five Scores

The prognostic significance of the Child-Pugh score, the MELD score, the MELD-Na score, the iMELD score, and the ALBI score calculated for 28-day, 90-day, and 6-month survival is summarized in Table 3. All prognostic scores showed significance in predicting mortality at 28 days, 90 days, and 6 months (*P* < 0.001). At 28 days, the ALBI score had the highest AUROC (0.714, 95% CI: 0.637-0.795), and the AUROCs of the Child-Pugh score, the MELD score, the MELD-Na score, and the iMELD score were 0.680 (95% CI: 0.619-0.763), 0.691 (95% CI: 0.621-0.785), 0.666 (95% CI: 0.573-0.759), and 0.681 (95% CI: 0.606-0.778), respectively. When predicting 90 days, the MELD score had the highest AUROC (0.711, 95% CI: 0.641-0.798) compared to the Child-Pugh score (0.663, 95% CI: 0.528-0.728), the MELD-Na score (0.707, 95% CI: 0.636-0.790), the iMELD score (0.712, 95% CI: 0.638-0.796), and the ALBI score (0.663, 95% CI: 0.589-0.738). The AUROCs of the Child-Pugh score, the MELD score, the MELD-Na score, the iMELD score, and the ALBI score are 0.679 (95% CI: 0.613-0.744), 0.723 (95% CI: 0.652-0.789), 0.703 (95% CI: 0.637-0.772), 0.713 (95% CI: 0.641-0.779), and 0.693 (95% CI: 0.630-0.767), respectively. All prognostic scores showed significance in predicting mortality at 28 days, 90 days, and 6 months (*P* < 0.0001). The AUROCs of the ALBI score at 28 days and the MELD score at 90 days and 6 months exceeded 0.700.

### 3.4. Comparing the Predicting Performance of the Five Scores

When assessing the prognostic performance of all five scores in terms of 28-day mortality, only the AUROC of the ALBI score was higher than 0.700, which shows moderate accuracy for predicting 28-day mortality; however, the AUROCs of the ALBI score at 90 days and 6 months were lower than that of the MELD score, which was less than 0.700. When assessing the prognostic performance of all five scores in terms of 90-day and 6-month mortality, the AUROCs of the MELD score, the MELD-Na score, and the iMELD score were higher than 0.700, and the AUROC of the MELD score was higher than that of the MELD-Na score and the iMELD score. At the 28-day, 90-day, and 6-month follow-up, the AUROC of the iMELD score was higher than that of the MELD-Na score. No significant differences were found among all five scores (*P* > 0.05). Comparisons of the AUROC of five scores are shown in Figure 1.

## 4. Discussion

Prognosis is an important part of any disease assessment. However, the prognostic information for specific patients is often unsatisfactory and plagues the clinic because the actual situation of the individual is often different from the average population on which the prognosis score is based. The source of diversity is mainly the patient's disease stage, etiology, and complications [23–25]. To eliminate the effect of disease stage and seek out a widely used and accurate score, patients with decompensated cirrhosis (DeCi) of this study were enrolled regardless of the cause of cirrhosis.

Decompensated cirrhosis is a common disease with high morbidity and may be accompanied by several manifestations of decompensation, including gastrointestinal hemorrhage, hepatic encephalopathy, and infection. Consistent with a previous study on patients with liver cirrhosis, approximately 11.0% of patients with decompensated cirrhosis died within 28 days and 20% died within 6 months in the present study [26–28]. To reduce mortality, it is crucial to recognize those patients with a potentially poor prognosis and then prioritize and treat them accordingly in an appropriate and timely manner. The Child-Pugh and MELD scores are the widely used scores for the assessment of liver function and serve as independently related factors for prognosis. Recently, the albumin-bilirubin (ALBI) score was used to assess liver function in DeCi patients. ALBI also has proven to be an independent predictor of survival in patients with DeCi [14]. To our knowledge, although the predictive significance of these scores for predicting survival in DeCi patients has been demonstrated, different conclusions have been made regarding the better predicting value of the Child-Pugh score versus the MELD score in DeCi patients [27, 29–31]. Due to the population characteristics and observation time of study, finding an optimal scoring standard is still a challenging issue.

As expected, the Child-Pugh score, the MELD score, and the ALBI score were associated with outcome and had a predictive value for 28-day, 90-day, and 6-month mortality. Then, by comparing the prognostic performance of the five scores at 28 days, the AUROC of the ALBI score was higher than that of the other scores. The ALBI score was originally used to assess liver function in patients with hepatocellular carcinoma and contains only two simple parameters, albumin and bilirubin [22]. The level of albumin and bilirubin can reflect liver function, and the change of albumin and bilirubin levels often means liver dysfunction and poor prognosis in patients with cirrhosis. Compared with the other scores, the ALBI score involves only two common continuous parameters that are easily acquired in clinical practice and are simply calculated by applying a formula. By studying 1067 cirrhotic patients, Shao et al. revealed that the ALBI score has a similar predictive efficiency for assessing the in-hospital death of patients with liver cirrhosis [32]. Lei et al.'s study shows that ALBI scores are consistent with the Child-Pugh score and the MELD scores in predicting value of patients with hepatitis B-related liver disease [14]. Similar to the conclusion of Xavier et al.'s study, we found that the ALBI score has a better performance than the Child-Pugh score and the MELD scores in predicting short-term prognosis, especially in patients with acute decompensation of cirrhosis [28]. Xavier et al.'s study mainly focused on patients with cirrhosis complicated by acute upper gastrointestinal bleeding, which is similar to the cause of hospitalization in this study. However, Xavier et al.'s research population were European Portuguese and the etiology of cirrhosis was not described. Chen et al.'s study concluded that the ALBI score is more accurate than the Child-Pugh and MELD scores for 3-month prognosis in hepatitis B-related cirrhosis patients, and Wang et al.'s study indicated that the prognostic performance of the ALBI score was superior to that of the MELD and MELD-Na scores for long-term outcomes [13, 33]. In our study, the predictive value of the ALBI score was lower than that of the MELD score, which implicated the important role of cirrhosis decompensation. When evaluating the predictive value of the scores for 90-day and 6-month survival, the AUROC of the MELD score was higher than that of the other scores, including the derivatives of the MELD score (MELD-Na, iMELD). In a previous study, there was much controversy about the predictive efficiency of the MELD and Child-Pugh scores for long-term outcomes [29, 31, 34–37]. The inconsistency of the study's conclusions was mainly due to the cause of cirrhosis, study population, and follow-up time. The prognostic assessment of patients with DeCi remains a challenging clinical issue. Therefore, new or adjusted scoring systems often were created. The Child-Pugh score is widely used in the clinic since it was proposed 50 years ago, and it is determined by calculating serum bilirubin and albumin, prothrombin time, hepatic encephalopathy, and ascites [8]. The presence or absence of ascites and hepatic encephalopathy, as part of the Child-Pugh score, contains significant subjectivity and has no clear cut-off value. The MELD score incorporates only 3 laboratory variables: bilirubin, INR, and creatinine; it is susceptible to diuretics, hemorrhage, and ascites, with an absence of clearly defined cut-off values for categorizing cirrhotic patients [38]. Most of the studies on the MELD score have been concentrated in Western countries, where the main cause of cirrhosis is alcoholic cirrhosis [6, 39, 40]. Whether the MELD score is suitable for the Asian population needs more research. A meta-analysis compared the prognostic performance of the Child-Pugh and MELD scores and concluded that they show similar prognostic significance with moderate discrimination. In specific circumstances, one of the scores has better predicting value than the other, such as the MELD score, which has better predictive value for critically ill cirrhotic patients [27]. In our study, one of the reasons why the predictive value of the MELD score was superior to that of the Child-Pugh score may be the objective index of creatinine that is associated with the mortality of DeCi patients [41]. Another reason for the higher predictive value of the MELD score may be the cause of cirrhosis. Hyponatremia and age are also important factors affecting the prognosis of patients with cirrhosis; therefore, some scoring systems derived from the MELD score have been created, such as the MELD-Na and iMELD scores [12, 21, 42]. The MELD-Na and iMELD scores not only consider liver and kidney function as well as etiology but also consider the electrolyte condition. The ability of the serum sodium level and age to evaluate the prognosis of DeCi patients compensates for the deficiency of the MELD score [43–45]. In this study, the AUROCs of the MELD-Na and iMELD scores were lower than that of the MELD score, which is inconsistent with the expected results. Inconsistent conclusions may be associated with serum sodium levels, which are susceptible to therapeutic intervention, leading to unstable reliability for long-term prognosis predictions. Another reason for the inconsistent conclusions may be related to the research population since most hospitalization causes were gastrointestinal hemorrhage, which differs from other research populations mainly based on complications of ascites and infection.

This study also has several limitations. First, as a single-center retrospective cohort study, the study may have a hereditary limitation, and some patients were lost to follow-up, which may have resulted in selection bias. Large multicenter, prospective studies are needed to test and verify our findings. Second, the scores were merely determined at admission, so we were not able to evaluate the dynamic predictive role of the scores. Finally, organ failure-related scores, such as the sequential organ failure assessment (SOFA) score and chronic liver failure consortium acute-on-chronic liver failure score (CLIF-C ACLFs) [46], were not detected. Furthermore, the correlation between these scores and lactic acid was not analyzed.

In summary, although there are many discussions and controversies on the predictive value of all kinds of prognostic scores, our results indicate that the Child-Pugh score, the MELD score, the MELD-Na score, the iMELD score, and the ALBI score are optimal tools for predicting the prognosis of patients with DeCi in China. The ALBI score has better predicting value for the assessment of short-term outcomes, and the MELD score has better predicting value for long-term outcomes, which can help to prioritize patients and guide clinicians in making appropriate treatment decisions.

## Figures and Tables

**Figure 1:** Comparisons of the receiver operating characteristic curves of the scores. MELD: model for end-stage liver disease; MELD-Na: MELD combined with serum sodium concentration; iMELD: integrated MELD; ALBI: albumin-bilirubin score. (a) ROC for 28 days; (b) ROC for 90 days; (c) ROC for 6 months.

**Table 1:** Characteristics of patients in the DeCi cohort.

Variable	Patients with decompensated cirrhosis (*n* = 456)
Sex (male), *n* (%)	344 (75.4%)
Age, median (IQR)	53.5 (46-63.75)
Hospitalization days, median (IQR)	11 (9-13)
Intensive care unit (%)	64 (14.0%)
Cause of liver cirrhosis, *n* (%)	
Viral	276 (60.5%)
Alcoholic	72 (15.8)
Combined alcoholic viral	37 (8.1%)
Other	28 (6.1%)
Cryptogenic	43 (9.4%)
Cause of hospitalization, *n* (%)	
Ascites	3 (0.7%)
Gastrointestinal hemorrhage	407 (89.2%)
Hepatic encephalopathy	22 (4.8%)
Infection	24 (5.3%)
Ascites degree, *n* (%)	
No ascites	195 (42.8%)
1st-degree ascites	123 (27.0%)
2nd-degree ascites	80 (17.5%)
3rd-degree ascites	58 (12.7%)
Renal failure, *n* (%)	20 (4.4%)
Hepatocellular carcinoma, *n* (%)	56 (12.3%)
Acute decompensation, *n* (%)	436 (95.5%)
Therapy, *n* (%)	
Vasopressor support	144 (31.6%)
Mechanical ventilation	27 (5.9%)
Renal replacement therapy	2 (4.4%)
28-day outcome, *n* (%)	
Lost to follow-up	31 (6.8%)
Survivors	375 (82.2%)
Nonsurvivors	50 (11.0%)
90-day outcome, *n* (%)	
Lost to follow-up	77 (16.9%)
Survivors	300 (65.8%)
Nonsurvivors	76 (16.6%)
6-month outcome, *n* (%)	
Lost to follow-up	132 (28.9%)
Survivors	233 (51.1%)
Nonsurvivors	91 (19.9%)

IQR: interquartile range.

**Table 2:** Comparison between the survival group and the nonsurvival group at the 28-day, 90-day, and 6-month follow-ups.

Parameter	28 days			90 days			6 months		
	Survivors	Nonsurvivors	*P* value	Survivors	Nonsurvivors	*P* value	Survivors	Nonsurvivors	*P* value
ALT (IU/l)	26 (18-42)	25.5 (15.75-56)	0.512	25 (17-38.25)	27 (16-54.75)	0.114	23 (17-36)	26 (15-56)	**0.040**
AST (IU/l)	40 (28-68)	67.5 (38.25-168.25)	**<0.001**	38 (26-57)	64.5 (36.5-160.25)	**<0.001**	35.5 (26-53)	58 (36-168)	**<0.001**
Albumin (g/l)	28.8 (25.4-31.4)	25.05 (21.75-28.575)	**<0.001**	29 (25.8-32)	25.65 (22.8-29.275)	**<0.001**	29.1 (25.925-32.1)	25.7 (22.8-29.5)	**<0.001**
Bilirubin (mmol/l)	23.8 (15.5-39.9)	36.2 (21.125-73.425)	**0.028**	22.85 (14.85-38.7)	27.1 (17.75-58.25)	**0.022**	21.9 (14.3-37.475)	29.5 (19.6-57.2)	**0.004**
ALP (IU/l)	70 (53-101)	115 (68.25-175.5)	**<0.001**	68 (53-96)	98.5 (67.75-167)	**<0.001**	67 (51.25-92.75)	95 (67-168)	**<0.001**
GGT (IU/l)	23 (14-56)	38.5 (18-128.75)	**0.020**	21.5 (13.75-47.25)	38 (21-106.75)	**<0.001**	21 (13-48)	37 (17-106)	**0.003**
Creatinine (mmol/l)	72.4 (59.6-91.3)	92.55 (72.65-134.35)	**<0.001**	72.3 (59.525-88.875)	92.55 (64.05-135.88)	**<0.001**	71.45 (57.7-86.075)	91.9 (63.4-132.6)	**<0.001**
INR	1.31 (1.2-1.5)	1.48 (1.24-1.95)	**<0.001**	1.3 (1.18-1.483)	1.425 (1.27-1.75)	**<0.001**	1.31 (1.19-1.487)	1.4 (1.24-1.76)	**<0.001**
PT	14.7 (13.5-16.7)	15.1 (13.7-21.45)	**0.002**	14.65 (13.175-16.425)	15.6 (13.825-19.9)	**<0.001**	14.7 (13.025-16.4)	15.4 (13.7-19.9)	**<0.001**
Platelet (10∗9/l)	62 (41-96)	74 (28.25-115.5)	0.893	62 (40.75-92.25)	69 (32.25-108)	0.637	64 (41-92.75)	70 (37-109)	0.419
WBC (10∗9/l)	6.34 (3.95-9.48)	9.37 (4.648-14.973)	**<0.001**	6.33 (3.865-9.05)	8.15 (4.715-13.63)	**0.001**	6.295 (3.805-9.432)	7.75 (4.42-13.57)	**0.003**
Na (mmol/l)	138.4 (136-141)	140.15 (134.45-143.88)	0.168	138.95 (136-141)	138.45 (134.85-142.75)	0.939	138.6 (136-141.15)	138.5 (135-142)	0.967
Child-Pugh score	8 (7-10)	10 (8-11)	**<0.001**	8 (7-9)	9 (8-10.5)	**<0.001**	8 (7-9)	9.5 (8-11)	**<0.001**
MELD score	11 (9-14)	15 (11-23)	**<0.001**	10.5 (9-14)	15 (11-20)	**<0.001**	10 (9-14)	14 (11-19.5)	**<0.001**
MELD-Na score	12 (9-15.410)	16 (12.295-25)	**<0.001**	11 (9-15)	15 (11.59-23)	**<0.001**	11 (9-14)	15 (11.59-22.837)	**<0.001**
iMELD score	30.695 (27.1-35.578)	37.14 (30.335-42.35)	**<0.001**	30.3 (26.53-34.1)	35.9 (29.72-42.2)	**<0.001**	30.17 (26.568-34.265)	36.1 (29.72-41.9)	**<0.001**
ALBI score	-1.541 (-1.813~-1.140)	-1.031 (-1.507~-0.449)	**<0.001**	-1.548 (-1.851~-1.177)	-1.140 (-1.544~-0.635)	**<0.001**	-1.553 (-1.886~-1.228)	-1.152 (-1.562~-0.652)	**<0.001**

Data are expressed as the median (interquartile range). ALT: alanine aminotransferase; AST: aspartate aminotransferase; GGT: gamma-glutamyl transpeptidase; INR: international normalized ratio; PT: prothrombin time; WBC: white blood cell count; MELD: model for end-stage liver disease; MELD-Na: MELD combined with serum sodium concentration; iMELD: integrated MELD; ALBI: albumin-bilirubin score.

**Table 3:** Predictive value of the prognostic scores calculated for 28-day, 90-day, and 6-month survival.

Prognostic score	AUROC	Asymptotic sig	Cut-off point	Sensitivity (%)	Specificity (%)	PLV	NLV
*28-day mortality*							
Child-Pugh score	0.680	**<0.0001**	14	77.30	52.00	1.61	0.44
MELD score	0.691	**<0.0001**	9	74.86	58.00	1.78	0.43
MELD-Na score	0.666	**<0.0001**	19.40	89.37	40.82	1.51	0.26
iMELD score	0.681	**<0.0001**	34.22	71.08	64.00	1.97	0.45
ALBI score	0.714	**<0.0001**	-1.168	73.17	64.00	2.03	0.42
*90-day mortality*							
Child-Pugh score	0.663	**<0.0001**	8	62.96	62.82	1.69	0.59
MELD score	0.713	**<0.0001**	12	66.67	67.95	2.08	0.49
MELD-Na score	0.707	**<0.0001**	14.95	78.26	54.12	1.71	0.40
iMELD score	0.712	**<0.0001**	34.10	74.29	65.12	2.13	0.39
ALBI score	0.693	**<0.0001**	-0.997	85.86	62.82	2.31	0.23
*6-month mortality*							
Child-Pugh score	0.679	**<0.0001**	8	64.76	63.95	1.80	0.55
MELD score	0.723	**<0.0001**	12	67.62	67.44	2.08	0.48
MELD-Na score	0.703	**<0.0001**	14.95	78.26	64.94	1.86	0.41
iMELD score	0.713	**<0.0001**	34.10	74.29	65.12	2.13	0.39
ALBI score	0.693	**<0.0001**	-1.188	79.15	54.65	1.71	0.41

MELD: model for end-stage liver disease; MELD-Na: MELD combined with serum sodium concentration; iMELD: integrated MELD; ALBI: albumin-bilirubin score; PLV: positive likelihood ratio; NLV: negative likelihood ratio.

## Data Availability

The data used to support the findings of this study are available from the corresponding author upon request.

## Supplementary Materials

Supplementary Materials Supplement Table 1: cause of death of patients with DeCi. Supplementary Table 2: basic information and treatment differences between those who were lost to follow-up and the overall patient.
